The article "Bioinformatics Analysis of Prognostic Significance and Immune Characteristics of CXC Chemokine Family in Patients with Lung Adenocarcinoma" was published in 2022. Journal: Comput Math Methods Med.

# Bioinformatics Analysis of Prognostic Significance and Immune Characteristics of CXC Chemokine Family in Patients with Lung Adenocarcinoma

**DOI:** 10.1155/2022/3918926

**Published:** 2022-07-06

**Authors:** Dachen Bian, Yanhua Chen

**Affiliations:** Department of Respiratory and Critical Care Medicine, Jiangsu Taizhou People's Hospital, Taizhou 225300, China

## Abstract

**Objective:**

To screen CXC chemokines related to the risk of lung adenocarcinoma (LUAD) using bioinformatics and construct a CXC-based prognostic risk model to improve the diagnosis and treatment of LUAD patients.

**Methods:**

The Cancer Genome Atlas (TCGA) database and Gene Expression Omnibus (GEO) database were searched to obtain mRNA expression data and clinicopathological information of LUAD patients. CXC genes differentially expressed in LUAD were screened using the R packages. Further, risk factors significantly associated with the survival of LUAD patients were obtained by the univariate Cox proportional hazard regression, LASSO regression, and multivariate Cox proportional hazard regression analysis, following which a risk prediction model was constructed. The performance of the CXCL13-based model in predicting the prognosis of low-risk and high-risk effect LUAD patients was verified, and the association between the model and the degree of tumor immune cell infiltration was investigated.

**Results:**

CXCL13 was significantly highly expressed in the cancer tissues of LUAD patients. The risk of death in patients with highly expressed CXCL13 was about 1.5 times higher than in those with lowly expressed CXCL13 (HR = 1.5153357). CXCL13-based risk scoring showed that the high-risk score of LUAD patients was significantly correlated with poor prognosis, but no relation between the two was found in the GEO validation sets, suggesting that this risk model may not be accurate enough. In addition, activated B cells, CD4+ T cells, CD8+ T cells, and dendritic cells were significantly positively correlated with the high risk of LUAD.

**Conclusions:**

Although we found that a high expression of CXCL13 was associated with a high risk of death and immune cell infiltration and activation in LUAD patients, the CXCL13-based risk model was not accurate enough for predicting the prognosis of LUAD patients.

## 1. Introduction

Lung cancer is by far the leading cause of cancer death in men and women, and approximately a quarter of cancer cases die of lung cancer [1]. According to different histological subtypes, it is divided into lung adenocarcinoma (LUAD), squamous carcinoma, large cell carcinoma, and small cell lung cancer [2], with LUAD as the most prevalent subtype [3]. In recent years, with the application of multimodal treatment strategies, including diagnosis, immunotherapy, molecular therapy, radiotherapy, and noninvasive surgical resection, the clinical prognosis of LUAD patients has improved significantly, but the five-year overall survival rate is still unsatisfactory at only about 18% [4, 5]. Currently, there is no ideal biomarker for various tumors, including lung cancer. Thus, comprehensive analysis of epidemiological and clinical data, molecular detection of blood biomarkers, tumor cell and tumor immune cell infiltration, and other analyses are required to obtain a more objective and accurate diagnosis and prognosis prediction [6].

The chemokine superfamily, composed of approximately 50 endogenous chemokine ligands and 20 G-protein-coupled receptors, is a class of small molecular weight proteins secreted by cells that regulate the function of the immune system. Their main roles are to regulate processes such as cell migration, localization, proliferation, differentiation, and survival. Additionally, they mediate development, homeostasis, and angiogenesis and participate in autoimmune diseases, inflammation, and tumor development [7–9]. According to the number and spacing of conserved cysteine residues in the N-terminus, chemokines can be classified into four categories: CC chemokines, CXC chemokines, C chemokines, and CX_3_C chemokines (X is other amino acid residues) [6, 8].

CXC chemokine subfamily is made up of 17 members (CXCL1–CXCL17). Studies have shown that multiple CXC chemokines play an important role in the malignant behaviors, including cancer development and cancer drug resistance, in various cancers such as glioma [10], leukemia [11], gastric cancer [12], colorectal cancer [13], and lung cancer [14]. However, it is unclear whether CXC chemokine subfamily members have some role in LUAD. Therefore, with LUAD patient data from the TCGA and GEO public databases, this study used differential analysis, univariate Cox regression, LASSO regression, and multivariate Cox regression to screen CXC chemokine subfamily members associated with LUAD. A prognostic risk model was then established based on the screened CXC genes, and the correlation between the model and tumor-infiltrating immune cells in LUAD patients was assessed.

## 2. Materials and Methods

### 2.1. Source of Data

Raw RNA-seq data and clinicopathological information of LUAD patients were obtained from the TCGA database (https://www.cancer.gov/), while the GEO database (http://www.ncbi.nlm.nih.gov/geo/) provided gene expression data of GSE31210 and GSE72094 datasets, with the former as the training set and the latter as the validation set.

### 2.2. Data Processing and Screening of Differentially Expressed Genes

The data were read using the R software (version 4.0.5). The datasets were normalized using the “limma” package, and differentially expressed genes (DEGs) in LUAD tissues and paracancerous tissues were screened. The significance of gene expression differences between two kinds of tissues was analyzed by *t*-test and ∣ logFC  | >1. *P* < 0.05 served as the cut-off criteria.

### 2.3. GO and KEGG Functional Enrichment Analyses

The biological functions of DEGs and the related signaling pathways were identified using GO and KEGG analyses. GO analysis, including biological process (BP), cellular component (CC), and molecular function (MF), and KEGG pathway enrichment analysis were performed using the DAVID online website (https://david.ncifcrf.gov/) [15]. *P* < 0.05 was considered as the threshold for statistical significance.

### 2.4. CXC Chemokine-Based Risk Prediction Modeling

#### 2.4.1. Univariate Cox Proportional Hazard Regression

CXC genes with expressions greater than the mean were labeled as high expression group and expressed as 1, while those with expression less than or equal to the mean as low expression group were expressed as 2. The univariate Cox proportional hazard regression analysis of CXC genes was performed using the coxph function in the R “survival” package to assess the relationship between LUAD-related CXC genes and overall survival (OS) of LUAD patients.

#### 2.4.2. LASSO Regression

LASSO is a penalized regression method that adjusts the regression coefficient with an L1 penalty and reduces the final weight of most potential indicators to zero, thereby decreasing the number of indicators with nonzero final weight [16]. LASSO regression analysis was performed using the glmnet function and cv.glmnet function of the R “glmnet” package, with the survival time (time) and survival status (status) as dependent variables and the expression levels of 14 CXC genes as independent variables. Such analysis aimed to screen for CXC genes associated with LUAD survival.

#### 2.4.3. Multivariate Cox Proportional Hazard Regression

The CXC genes obtained from screening by the LASSO regression and univariate Cox proportional hazard regression were then included in the multivariate Cox regression model. The obtained CXC genes with expression greater than the mean were labeled as high expression group and expressed as 1, while those with expression less than or equal to the mean as low expression group were expressed as 2. The multivariate Cox proportional hazard regression analysis of CXC genes was performed using the coxph function in the R “survival” package. The risk index of each sample was predicted according to regression coefficient *β*, and the calculation formula of the risk index was RiskScore = *Σβi*∗*xi*.

### 2.5. Validation of the Proportional Hazard Model

According to the formula RiskScore = 0.40333∗CXCL13, the risk score of TCGA LUAD training set (533 cases), GSE31210 (246 cases), and GSE72094 dataset (442 cases) samples was calculated. The risk score greater than the mean was marked as highRisk and those less than or equal to the mean as lowRisk. Survfit function and Surv function of R package “survival” were used for survival analysis and for drawing of the Kaplan-Meier (KM) survival curve and survdiff function for a log-rank test. Usage of roc.curve function with RiskScore as the marker values was applied to plot the receiver operating characteristic (ROC) curve and calculate the area under the ROC curve (AUC).

### 2.6. Construction of Prediction Nomogram

A prediction nomogram was constructed by integrating the age, gender, TNM stage, and risk score of LUAD patients in TCGA LUAD samples, thus predicting the relationship between each variable in the model and survival. A nomogram function of the R package “rms” was constructed and plotted to predict the 1-year, 2-year, and 3-year survival rates of LUAD patients.

### 2.7. Single-Sample Gene Set Enrichment Analysis

Single-sample gene set enrichment analysis (ssGSEA) was carried out using the gsva function of the R package “GSVA,” and the immune scores of the high-risk and low-risk groups were calculated to evaluate the degree of tumor immune cell infiltration.

## 3. Results

### 3.1. Differentially Expressed CXC Genes and GO and KEGG Enrichment Analyses

The clinical information and RNA-seq data of lung tissues from 594 LUAD patients, including 61 normal tissues and 533 cancer tissues, were downloaded from the TCGA database. The TCGA-derived mRNA sequencing data of LUAD patient tissues collated in this study matched CXC genes to obtain the expression of 14 CXC genes in lung tissue except for CXCL4, CXCL7, and CXCL15 (Figure 1(a)).

KEGG and GO analyses were then performed on these 14 CXC genes. GO analysis results showed that the 14 CXC genes associated with LUAD were mainly enriched in leukocyte chemotaxis, leukocyte migration, cell chemotaxis of BP (circular markers in Figure 1(b)), external side of the plasma membrane of CC (square markers in Figure 1(b)), and chemokine activity of MF (diamond markers in Figure 1(b)). KEGG analysis showed that the 14 CXC genes associated with LUAD were mainly enriched in signaling pathways such as chemokine pathway, cytokine-cytokine receptor interaction, viral protein interaction with cytokine, and cytokine receptor (triangular markers in Figure 1(b)).

By differential expression analysis of genes in adjacent noncancerous tissues and LUAD tissues with the cuff-off criteria of ∣ logFC  | >1 and *P* < 0.05, 1673 DEGs were obtained, including 679 upregulated genes (red scatters in Figure 1(c)) and 994 downregulated genes (green scatters in Figure 1(c)). The intersection of DEGs with 14 CXC genes by the Wayne diagram showed that 6 CXC chemokine genes had significantly abnormal expression in LUAD tissues, of which CXCL2, CXCL3, CXCL12, and CXCL16 were significantly downregulated in LUAD tissues, while CXCL13 and CXCL14 were significantly upregulated (Figure 1(d)).

### 3.2. Risk Prediction Model of CXC Genes in LUAD

The relationship between CXC chemokine genes and OS of LUAD patients was assessed by the univariate Cox proportional hazard regression. The results showed that among the 14 CXC chemokine genes expressed in LUAD, only the regression coefficient coef (beat value) of CXCL13 was statistically significant (*P* = 0.0014), indicating that LUAD patients with high CXCL13 expression had a higher risk of survival, and their risk of death was approximately 1.5-fold higher than of patients with low CXCL13 expression (HR = 1.52, Figure 2(a)). Further, LASSO regression was employed for screening CXC genes significantly associated with OS time and survival status of LUAD patients. The results revealed that none of the LASSO regression coefficients were 0. Three stable genes (CXCL6, CXCL5, and CXCL17) at the right side of the dashed line were selected as the optimal genes for modeling (Figures 2(b)–2(d)), suggesting that these three genes were significantly associated with the prognosis of LUAD patients. Finally, CXCL13, CXCL6, CXCL5, and CXCL17 were included in the multivariate Cox regression model. CXCL13 was found to be an independent risk factor for LUAD (*P* = 0.0194), with the coef of CXCL13 = 0.40333 and its risk score in LUAD being RiskScore = 0.40333∗CXCL13 expression.

### 3.3. CXC Gene-Based Establishment of Prognostic Characteristics and Validation of Their Predictive Performance

The risk score of the TCGA training set samples was calculated according to the risk score formula, with risk scores greater than the mean labeled as highRisk and those less than or equal to the mean labeled as lowRisk. The results showed that there were 160 patients in the highRisk group and 360 patients in the lowRisk group in the TCGA training set. Based on KM curves, high-risk patients had significantly worse OS rates than low-risk patients (Figure 3(a), *P* < 0.05). In addition, ROC curve analysis showed that the AUC of this risk model for the 1-year, 2-year, and 3-year survival prediction curves was less than 0.6, suggesting that the predictive value of this model for the real high and low risks of LUAD was unsatisfactory (Figure 3(b)). The GSE31210 and GSE72094 datasets were subsequently used as validation sets to validate the effect of the risk model. The results showed that the GSE31210 dataset contained 124 highRisk samples and 102 lowRisk samples, and the GSE72094 dataset contained 212 highRisk samples and 173 lowRisk samples. KM survival curves indicated that this risk model was not significantly associated with survival in LUAD patients in both GEO validation sets (Figures 3(c) and 3(d)*P* > 0.05). In addition, a nomogram was drawn based on clinical information such as age, gender, and TNM stage of TCGA LUAD patients and calculated risk scores to predict the 1-, 2-, and 3-year survival rates of LUAD patients (Figure 3(e)).

### 3.4. Levels of Infiltrating Immune Cells in Patients with High-Risk and Low-Risk LUAD

To clarify the relationship between the constructed risk prediction model and immune cell infiltration, we applied the ssGSEA method to the transcriptome of the TCGA LUAD samples to assess the immunity of different risk groups. Twenty-eight kinds of infiltrating immune cells were included to estimate the immune capacity of LUAD patients. The results showed that immune cells or immune processes such as activation of B cells, CD4+ T cells, CD8+ T cells, and dendritic cells were significantly and positively correlated with the high risk of LUAD patients (*P* < 0.01), and the correlation coefficient *R* reached 0.872 (Figure 4).

## 4. Discussion

Chemokines are important components of the tumor microenvironment and have multiple regulatory functions that can act on both the tumor microenvironment and tumor cells [6]. This study explored whether the CXC chemokine subfamily genes could serve as prognostic factors and could be used to construct effective risk models for LUAD patients. Upon differential analysis of CXC gene expression in LUAD patients from the TCGA LUAD, we found that the expression levels of CXC2, CXCL3, CXC12, and CXC16 in tumor tissues of LUAD patients were significantly lower than in normal tissues, while CXCL13 and CXC14 were significantly highly expressed in tumoral tissues compared to normal ones. Unlike our results, multiple studies have shown that CXCL2, CXCL3, CXC12, and CXC16 were highly expressed in lung cancer tissues and are essential for tumor growth [17–20]. However, the findings of Fan et al. were consistent with this present study [21]. Highly expressed CXCL13 and CXCL14 in lung cancer tissues were also reported in other studies [22, 23].

CXCL13, also known as B cell-attracting chemokine 1, is a homeostatic chemokine used to recruit B cells, a few T cells, and macrophages [24]. In recent years, CXCL13 has been proved to be expressed at high levels in various malignant tumor tissues such as gastric cancer [25], breast cancer [26, 27], colorectal cancer [28], lung cancer [29, 30], prostate cancer [31], and lymphoma and correlated with tumor size, stage, lymph node metastasis status [25], sex hormone levels, drug treatment response [32], and tumor recurrence. Collectively, CXCL13 is considered as a potential prognostic and therapeutic marker. It was reported that the overexpression of CXCL13 could promote the growth, migration, invasion, and epithelial-mesenchymal transformation of tumor cells [16]. Wang et al. found that CXCL13 was overexpressed in 62% of smokers and 45% of nonsmokers in lung cancer patients [29]. Animal experiments confirmed that CXCL13 was involved in the development of benzopyrene-induced lung cancer [29], and Singh et al. demonstrated significantly higher serum levels of CXCL13 in lung cancer patients compared with healthy controls [30]. Combining the above previous studies and the survival and prognosis data obtained from our study, it can be speculated that CXCL13 could be a potential prognostic marker for LUAD, and its expression level is significantly and negatively correlated with the survival of LAUD patients. Using the above prognostic analysis results, we further established a CXCL13-based risk prediction model. The performance of the model was validated using the mRNA expression of LUAD patients derived from the GEO datasets. However, the risk score based on CXCL13 expression level in the GSE31210 and GSE72094 datasets showed no significant correlation with the survival of LUAD patients (*P* > 0.05), and the AUC value of the ROC curve based on the TCGA LUAD data also suggested that the model had an unsatisfactory prediction accuracy of 1-year, 3-year, and 5-year survival of LUAD patients. Such results could be explained by the selection of TCGA and GEO original data.

Tumor immune infiltration analysis showed that a high level of CXCL13 and corresponding high risk of LUAD were positively correlated with the activation of B cells, CD4+ T cells, CD8+ T cells, and dendritic cells. As reported, CXCL13 and its receptor CXCR5 can enhance B cell receptor-mediated B cell activation [33]. In breast cancer patients, tumor-infiltrating CD4+ lymphocytes were shown to be a vital source of CXCL13 [34]. High levels of CXCL13 in patients with chronic hepatitis B stimulated the recruitment of CXCR5+ CD8+ T cells to produce high levels of HBV-specific interferon-*γ* and IL-21 in patients with chronic HBV infection to improve viral control [35]. CXCL13 mediates B cell recruitment in tumor tissues while being essential for the formation of tertiary lymphoid structures (TLSs), and CXCL13+ CD103+ CD8+ TILs may play a critical role in mediating B cell recruitment and TLS formation in human tumors [36]. Animal experiments by McDonald et al. showed that dendritic cells could produce CXCL13 and participate in the development of small intestinal lymphoid tissue [37]. Taken together, we speculate that the high level of CXCL13 in cancer tissues of LUAD patients may be related to the activation and recruitment of B cells and T cells, and B cells and dendritic cells may be important sources of CXCL13.

This study still had some limitations. All the results of this study were based on bioinformatics calculations and were not verified experimentally. Also, the algorithm may have screened out some important prognostic factors.

## 5. Conclusions

In summary, CXCL13 was found to be significantly and highly expressed in LUAD tissues compared to normal tissues. Based on the risk assessment, CXCL13 was an independent risk factor for LUAD and was significantly associated with poor prognosis in LUAD patients. However, its predictive model failed to provide accurate results in the GEO database. In addition, activation of B cells, CD4+ T cells, CD8+ T cells, and dendritic cells were also found to be positively correlated with high risk in LUAD patients (*R* = 0.872).

## Figures and Tables

**Figure 1:** Differentially expressed CXC genes and GO and KEGG enrichment analyses. (a) Wayne diagram showing LUAD-related CXC chemokine genes in the TCGA dataset. (b) GO analysis and KEGG analysis of LUAD-related CXC chemokine genes (abscissa GeneRatio is the ratio of the number of genes enriched in each item to the total number of differential genes, that is, the enrichment; the more rightward the marker, the higher the enrichment). (c) Screening of DEGs in LUAD tissues in the LUAD TCGA dataset and visualization by volcano plot. (d) Wayne diagram of CXC chemokine genes significantly differentially expressed in LUAD tissues.

**Figure 2:** CXC chemokine-based risk prediction modeling for LUAD. (a) Univariate Cox proportional hazard regression analysis to assess the relationship between CXC genes and overall survival in LUAD patients, ^∗∗^*P* < 0.01. (b and c) Prognostic characteristics constructed by the minimum criteria of the LASSO Cox regression algorithm, with each curve representing the change trajectory of each independent variable coefficient (b); the corresponding genes at the site of the dashed line which was marked as the minimum value of log *λ* were the optimal genes for modeling (c). (d) Multivariate Cox proportional hazard regression analysis based on the risk score formula.

**Figure 3:** CXC gene-based establishment of prognostic characteristics and validation of their predictive performance. (a) Kaplan-Meier survival curve to assess the prognostic value of the risk model for LUAD patients. (b) AUC of the risk model for the 1-year, 2-year, and 3-year survival prediction curves. TP represents TRUE positive, and FP is FALSE positive according to cutoff. (c and d) GSE31210 dataset (c) and GSE72094 dataset (d) used to validate the predictive performance of the risk model for survival of LUAD patients. (e) A nomogram constructed based on the risk score of the TCGA LUAD training set and the clinical characteristics of the patients.

**Figure 4:** Relationship between LUAD risk prediction model and infiltrating immune cells/processes. Specifically, ssGSEA was performed to investigate the correlation between LUAD risk and 28 immune-related cells/processes.

## Data Availability

The data used to support the findings of this study are available from the corresponding author upon request.
